The article "An Analysis of the Effects of the English Language and Literature on Students' Language Ability from a Multidimensional Environment" was retracted in 2023. Reasons: signs of a paper mill; suspected computer-generated content; unreliable results or conclusions; lack of ethics approval or compliance.

# An Analysis of the Effects of the English Language and Literature on Students' Language Ability from a Multidimensional Environment

**DOI:** 10.1155/2022/3225096

**Published:** 2022-09-13

**Authors:** Weifang Chen

**Affiliations:** Department of Public Basic Courses, Hunan Environment-Biological Polytechnic, Hengyang 421005, China

## Abstract

One of the most crucial components of a student's language proficiency is basic language proficiency, which is also its fundamental component. The development of students' language skills is greatly aided by ELL (English Language and Literature). It can not only foster the growth of students' language thinking but also widen their perspectives and enhance their capacity for language comprehension. In this essay, the rules of English are examined from the multifaceted ELL viewpoint. This study extracts personality characteristic data from practical texts and incorporates it into a modelling process of students' knowledge changes based on DM- (data mining-) related technology and multidisciplinary expertise. According to the *t*-test results, ELL, which incorporates communicative competence, has started to take on a role in education and is helping students' language skills. The performance gains are 3.95, 4.21, and 3.66, when the number of computing nodes is increased to 10, 20, and 30 times that of the original nodes, and the linear expansion indices are 0.914, 0.928, and 0.93. This proves that the Hadoop+Hive-based data cleaning tool has excellent linear scalability.

## 1. Introduction

As a tool of emotional expression between people, language has important value. With the common development of the world economy, politics, and culture, English is widely used in political, economic, and cultural exchanges. The ultimate goal of ELL (English Language and Literature) learning is to cultivate students' ability of listening, speaking, reading, and writing in English subjects, so as to promote the all-round and healthy development of students' comprehensive English language literacy. Through the study of human core instinct, we can analyze and understand human nature with the help of spoken, written, and even sign languages [1]. As a widely used language in the world, English plays an important role in easing conflicts and promoting ethnic exchanges. At this stage, the study of English is no longer limited to the superficial level of communication and communication. The research work of ELL should focus on the combination of the English language and other disciplines, as well as the problems between depth and breadth.

With the continuous development of social culture, the research work of ELL is getting deeper and deeper. At this stage, English is not only the basic aspect of language but researchers need to pay more attention to the integration and development of English with other disciplines. To help students swiftly grasp the abilities of listening, speaking, reading, writing, and translating and use them in their daily lives, this course is aimed at educating students on the background of English literature and its historical development. The use of a multidimensional perspective, according to the available research, can better enhance the advancement and development of our nation's ELL [2]. According to several studies [3], linguistic research should not only examine language behavior but also foster language proficiency and transform it into language application practice, dismantle disciplinary boundaries, and widen research horizons—that is, apply multidimensional viewpoints. Through the language scope, language teaching, language communication, and application classification, students receive all-around language instruction during the teaching process, enabling them to acquire English language information and improve their English language proficiency. In order to enhance students' overall English language proficiency, it places a strong emphasis on developing students' comprehension and practical application of English as well as how to use it successfully in both daily life and academic pursuits.

English communication ability is also an important part of students' language ability [4]. Of course, only when students have a certain basic knowledge of language can they cultivate a certain English communication ability. The application of multidimensional perspective can serve the exploration of our country's ELL and promote the overall progress and development of our country's ELL. Based on the multidimensional perspective, this study explores the contradiction between language input and output in college English writing in order to improve students' English writing ability. ELL will gradually connect with other disciplines to form a wider interdisciplinary research system and provide better services for human life practice. Therefore, it is feasible to study ELL from a multidimensional perspective.

### 1.1. Research innovation

1. Based on the multidimensional perspective, the oral English classroom model guided by constructivism is used for teaching and literature survey, questionnaire survey, test, and interview are used as the research methods
2. Using DM-related technology and multidisciplinary knowledge as the method and theoretical basis, aiming at the complexity and variability of learning activities, a dynamic cognitive diagnostic analysis study was carried out. Mining the attribute and personality information at the text level and integrating it into the students' knowledge change the modeling process

## 2. Related Work

### 2.1. Studies Related to English Teaching

Fernanda and Cristiane proposed that in order to implement the task-based teaching method in classroom teaching, the corresponding task-based test standard for teacher evaluation should be introduced [5]. The teaching activity design of the Seo task-based teaching method is explored in practice [6]; Macaro et al. implement task-based teaching in class, which can stimulate students' enthusiasm and interaction in learning English and cultivate their English application ability [7]. Nicholas' research found that teachers cannot accurately grasp the students' nearest development zone because they strictly follow their own curriculum and do not participate in the teacher-student interaction adjustment, which leads to students' language learning failure or learning confusion [8].

Groves and Mundt gave “the model, method, and design of constructivist teaching.” It is proposed that the center of the constructivist teaching mode is learners and learners, as the core of cognition, construct knowledge and construct meaning [9]. Warner and Dupuy did research and thinking on teaching Chinese as a foreign language based on constructivism theory. On the premise of analyzing a large amount of data, this paper summarizes the present situation of constructivism in foreign language teaching [10]. Howlett and John think that lexical chunks are a patterned language structure, stored in the human brain as a whole, and are the smallest and most ideal unit of communication and language processing [11].

### 2.2. Research Status of DM

As an important step in the process of knowledge discovery, DM (data mining) has the ability to discover useful patterns hidden in general data. The idea of DM draws lessons from other fields such as machine learning, pattern recognition, statistics, database system, and data visualization. There are specific premises and restrictions, specific to the domain and easy for users to understand.

Bagui et al. transformed the FP-growth algorithm into the MapReduce algorithm and proposed the PFP-growth algorithm, which proved that this algorithm has strong expansibility and is suitable for sea volume DM [12]. Xia et al. pointed out that with the increasing scale of datasets in the real world, when mining association rules, using existing algorithms, memory often becomes the bottleneck of execution, resulting in a lot of association rule mining work being impossible [13]. Zheng et al. conducted in-depth research on the problems and solutions in the mining process. There are many foreign achievements in the research of parallel association rules of mining, and a lot of successful technologies and experiences have been accumulated [14].

Based on database decomposition, Lee et al. suggested a new approach for mining association rules. Numerous useful systems have been created on this foundation [15]. According to Van Woezik and others, formative evaluation is more crucial to students' learning than summative evaluation. They also understand that giving students prompt feedback and formative evaluation can pique their interest and encourage further learning [16]. We can intuitively comprehend the classification criteria when using the Wood (decision tree) algorithm for classification, which is a classification approach with quick speed, high accuracy, simple generation mode, understandability, and consistency with human thinking and decision [17]. According to Man et al. [18], regression analysis may predict the prediction target and views the prediction attribute as an independent variable.

## 3. Methodology

### 3.1. DM in Formative Assessment of Language Learning

The language environment has a direct impact on English language communication. Language communicators express their language communication through the changes of different language environments, which is called language communication skills. In English language teaching, the language that accurately describes things can be regarded as the object of philosophical investigation. In the process of practical use, the meanings expressed by different language structures can be reflected. Therefore, according to the theory of contradiction, in the scientific system, ELL and other disciplines should not be isolated and independent development models, but interrelated R&D models, thus promoting the further development of ELL. In the process of English language practice, it is necessary to closely integrate with other related disciplines and to maximize the effect of ELL analysis and exploration by combining them.

Compared with classroom teaching, using video can make students see and hear correct pronunciation movements and mouth shapes better and correct past wrong pronunciation habits. That is, through explicit feedback and structured input exercises, the learners' internal input processing program is optimized, and then, the correct collinear connection between the grammatical form and meaning is formed in the learners' working memory but the psychological recognition and meaning in the process of connecting forms are not understood. Analyze the limitations of knowledge and the mechanism of language learning. Language often represents a person's psychological activities and behaviors, and political decisions of all countries are expressed through language. Therefore, researchers should pay attention to the study of language from a political point of view and study different language developments according to the development of different periods.

In ELL, no matter what kind of work you are engaged in, the basic knowledge of English language application, grammar knowledge, using skills, and language rhetoric are spread to a certain extent. In the process of reading, students can not only experience the knowledge conveyed by the article but also have a deeper understanding of the application skills of knowledge points, the use of rhetorical devices, vocabulary, and grammar. All students' knowledge will be expanded accordingly. Therefore, English teachers are needed to help students complete their ELL study, so as to improve their communicative competence.

Formative evaluation of learners in the process of language learning analyzes and extracts a lot of information left by learners in the learning process and provides timely, objective, and scientific information for learners according to the analysis. It is very important for both students and teachers to form sexual assessment and assessment feedback suggestions. Teachers can put forward appropriate suggestions or guidance according to students' formative evaluation to help them learn more effectively and improve the follow-up teaching effect.

Let *X*, *Y* be a pair of random variables. Their joint probability *P*(*X*⇒*x*, *Y*⇒*y*) refers to the probability that *X* takes the *x* value and *Y* takes the *y* value, while conditional probability *P*(*Y*|*X*) refers to the probability that one random variable *Y* takes a certain value when another random variable *X* has a known value. Formula (1) can be obtained as follows:

(1) $$\begin{array}{c} P\left(Y\left|X\right.\right)=\frac{P\left(X,Y\right)}{P\left(X\right)}=\frac{P\left(X\left|Y\right.\right)P\left(Y\right)}{P\left(X\right)}. \end{array}$$

The independence between attributes, often known as the Bayesian formula, is crucial for precise categorization. Additionally, it takes a lot of computing power to determine the Bayesian optimal hypothesis [19, 20]. The next generation of measurement theory is represented by cognitive theory. Its goal is to assess and analyze each student's level of microknowledge or their proficiency in various knowledge domains (such as functions and geometry). This is how the model is expressed:

(2) $$\begin{array}{c} P\left(X_{ji}=1\left|\theta_{j,s_{i},g_{i}}\right.\right)=g_{i}^{1-\pi_{ji}}s_{i}^{\pi_{ji}},\\ \pi_{ji}=\overset{K}{\underset{k=1}{\prod }}\theta_{jk}^{q_{ik}}. \end{array}$$

Among them, *K* represents the total number of knowledge and skills and {*g*_*i*_, *s*_*i*_} represents the “guess” factor and “mistake” factor in exercise *i*, respectively. *π*_*ji*_ indicates the mastery of exercise *i* by student *j*, which is influenced by student-knowledge vector *θ*_*j*_ and exercise-knowledge vector *q*_*i*_.

With the increase of the number of processors, the efficiency of the algorithm is seriously reduced due to the unbalanced load. Moreover, even with the optimal communication scheme, the communication cost will change linearly with the increase of the number of transactions. Given the example *x* of multiprocessor scheduling problem, the number of processors is *p*, and for any work sequence, the approximate solution with metric *m*(*x*) is found to satisfy the following:

(3) $$\begin{array}{c} \frac{m\left(x\right)}{m^{*}\left(x\right)}\leq \left(2-\frac{1}{p}\right), \end{array}$$

where *m*^∗^(*x*) is the measure of the optimal solution.

The intelligent teaching system model based on Web and DM mainly adopts DM technology. By analyzing a large amount of information accumulated on the website, it finds the patterns and rules that users are interested in, provides learning information for planners and managers, improves the course design, reconstructs site information, provides students with different learning contents according to their learning situation, and establishes a personalized and intelligent distance education environment. The model structure is shown in Figure 1 as follows:

Among them, the DM module is the key component to establish this open and intelligent distance learning environment, which mainly provides established models and rules for teachers and administrators by analyzing the data in the database. This module is mainly composed of four parts: preprocessing module, algorithm module, display module, and feedback module.

Under the current system, we mainly consider three aspects in evaluating students' cognitive ability: memory, understanding, and application. In the past, most teaching systems only considered the unilateral ability test of a given problem when evaluating cognitive ability. In order to objectively evaluate students' abilities in these three aspects, we have established corresponding weight levels for each question, including memory, understanding, and application. And constitute a capability weight matrix *R*_*ij*_ as follows:

(4) $$\begin{array}{c} R_{ij}=\left[\begin{array}{ccc} r_{11} & r_{12} & r_{13}\\ \vdots & \ddots & \vdots \\ r_{i1} & r_{i2} & r_{i3} \end{array}\right]. \end{array}$$

In this way, each cognitive ability score can be calculated by the following formula:

(5) $$\begin{array}{c} A_{j}=\frac{\sum_{i=1}^{m}t_{i}\cdot r_{ij}}{\sum_{i=1}^{m}r_{ij}}. \end{array}$$

Vocabulary is the foundation of language, as well as the foundation of language teaching and research. But it is not easy to define what a word is. From the actual effect, paying attention to students' state of affairs can make them learn knowledge in a pleasant environment and improve their language ability. Not every strategy is suitable for all learners, so the appropriate training strategy should be chosen according to the actual situation of each learner. The positive significance of strategy teaching is that it can cultivate students' autonomous learning ability and greatly improve learning efficiency.

### 3.2. Analysis of Improving Students' Language Ability from a Multidimensional Perspective

Adults have a wide variety of linguistic structures at their disposal, some of which can be categorized and others which cannot. It depends on whether the purposes or meanings of these structures are appropriate in the given situation. It is more beneficial for learners to repeatedly employ this relationship in linguistic input and output rather than only perceive it. Even if some grammatical forms are frequently written, they are nonetheless challenging to learn. This is due to the possibility that form and meaning will eventually align. This is largely related to the subject matter that pupils learn in their first language. Once the signal is blocked, learners will no longer be able to continuously learn the signal as they age, especially second language learners. Inattention is to blame for everything.

English learners know nothing about the learning content, learning objectives, and learning value of the ELL course. Therefore, it is particularly important to discuss and construct the curriculum objectives in the first class. The investigation and exploration of English itself are a process involving communication and cultural communication. Through the research and analysis of recent cognitive development, we can conclude that linguistics plays a vital role in the development of other related disciplines. Besides, neither English nor Chinese is the result of any combination. The more advanced the culture, the richer the cultural connotation of the language. Language expression focuses on the formation of internal rules according to national culture and customs. From a multidimensional perspective, through the above comparative analysis, we can find the differences between English and Chinese expressions and help students understand the meaning of English sentences correctly.

It can be seen that in real English communication, in order to express themselves accurately, students need to use different English rhetorical devices reasonably to help each other understand their intentions and achieve effective communication. Through reading and learning English literary works, on the one hand, students are provided with examples of written expressions, and on the other hand, they are allowed to learn English rhetorical skills and language expressions used in literary works. Therefore, strengthening the study of ELL is helpful to improve students' understanding of English, and at the same time, they can master more language skills, which is of great significance to improve their language ability and comprehensive quality.

In this study, due to the large amount of data of the mining object, limited by the research purpose and the time and space complexity of DM algorithm, it is necessary to select the relevant datasets and records, which have nothing to do with the pre-extraction problem. Make appropriate choices. When the total number of instances is small or large, the effects of these two sampling methods are basically the same. In order to avoid repeated sampling, this study uses random sampling without substitution. According to the sample size formula of random sampling without replacement,

(6) $$\begin{array}{c} n=\frac{z^{2}\left(p\left(1-p\right)\right)N}{\varepsilon^{2}N+z^{2}\left(p\left(1-p\right)\right)}, \end{array}$$

where *n* is the sample size based on the average, *N* is the number of instances of the dataset, *p* is the proportion of variables, *ε* is the error of the expected average sampling relative to the whole variable, and *z* is the confidence degree of the expected average sampling error. According to this, the sample size can be estimated.

When the dataset is decomposed into frequent itemsets, the candidate frequent itemsets also need to scan the original dataset to determine the frequent itemsets. For example, when the original dataset is decomposed according to the frequent binomial set, the number of candidate frequent binomial sets is usually very large and the original dataset needs to be scanned for counting, which also means that a large number of candidate frequent binomial sets will be stored in the decomposed dataset files. The sum generated on the disk is much larger than the original dataset.

Let the data point set in a cluster be *x*_*i*_ = {*x*_*i*1_, *x*_*i*2_,⋯,*x*_in_}^*T*^, *i* = 1, 2, ⋯, *N*, calculate the center point *μ* = (1/*N*)∑_*i*=1_^*N*^*x*_*i*_ and covariance matrix of the cluster, and get the Mahalanobis distance from the data point to the cluster center *μ* as follows:

(7) $$\begin{array}{c} d_{m}\left(x_{i},\mu \right)=\sqrt{{\left(x_{i}-\mu \right)}^{T}\overset{-1}{\sum }\left(x_{i}-\mu \right)}. \end{array}$$

The first-level frequent itemsets and second-level candidate sets are formed following the conclusion of the data initialization process. Based on this, all frequent itemsets will be iteratively generated during the iteration phase. The distribution of data nodes used to create the second-level frequent set is depicted in Figure 2. As you can see, there will be a significant bottleneck here because the second-tier candidate set is typically a large data collection. The candidate set can be selectively read in accordance with the traits of the transaction set to increase the effectiveness of this stage.

When the number of *k* is small, the process will consume a lot of resources. Through the analysis of the transaction set, it can be seen that the candidate set that the transaction set can contain must be the candidate set element between the first element of the transaction set and the last element of the transaction set, because the transaction set is in order. The elements of the transaction set are transferred to the frequent set and the corresponding ID in the order. At the same time, the items that do not belong to frequent set 1 are directly deleted to reduce the data volume of the original transaction set.

The decline in students' knowledge level over time is reflected in the students' recollection of that knowledge, which is deteriorating at an alarming rate. The two-parameter hyperbolic form is used to construct the memory factor because it has a more robust modelling effect than the hyperbolic form. Therefore, the memory factor *L*_*ik*_^*t*^(∗) can be defined as follows:

(8) $$\begin{array}{c} L_{ik}^{t}\left(*\right)=U_{ik}^{t-1}\frac{{Df}_{ik}^{t}}{f_{ik}^{t}+r}, \end{array}$$

where *f*_*ik*_^*t*^ represents the number of times that students learn related topics about knowledge concept *K* from *t* − 1 to *t*. *r*, *D* is a superparameter, which controls the amplitude and coefficient of knowledge level growth, respectively.

The goal of grade prediction is to predict students' grades for unanswered questions. Low prediction scores usually reflect students' familiarity with relevant knowledge concepts. Performance prediction is also the basis of personalized recommendation. Therefore, many online learning systems quantify students' learning process and show their knowledge evolution chart by learning behavior, so as to cultivate students' autonomous learning ability.

In order to find the optimal recommendation strategy *π*, the goal of the standard reinforcement learning algorithm is to learn the optimal action cost function *Q*^∗^(*s*, *a*), that is, take action *a* based on state *s* to maximize the expected return. The penalty is *γ* ∈ (0, 1), according to which the optimal action-value function satisfies the bellman equation:

(9) $$\begin{array}{c} Q^{*}\left(s,a\right)=\exists_{s^{\prime }}\left[r+\gamma \underset{a^{\prime }}{\max}Q^{*}\left(s^{\prime },a^{\prime }\right)\left|s,a\right.\right]. \end{array}$$

Compared with the topic set, the records of the topics that students have studied are very few, so this extremely sparse historical record also makes it very difficult to calculate the estimation of all state-action pairs step by step. Especially, when students have not done a topic, the algorithm cannot update the estimation of state transition to the new state based on the feedback of the topic.

All neurons in the same row compete with each other for the same input training vector, and the winning neuron adopts the winner-take-all strategy, so that its output is 1 and the output of other neurons in the same row is 0. That is, the input-output relationship of neurons in the same row is as follows:

(10) $$\begin{array}{c} V_{x,j}\left(t+1\right)=\left\{\begin{array}{c} 1,\;\text{if }j=m=\arg\left\{\underset{i}{\max}\left(U_{x,i}\left(t\right)\right)\right\},\\ 0,\;\text{if }j\neq m. \end{array}\right. \end{array}$$

Through the introduction of the competition mechanism, it can be ensured that the output of only one neuron in each row is 1, that is, the neuron that wins the competition. At the same time, it can also ensure that all *n* training vectors will be classified into class *c*. Moreover, the network can quickly converge to the minimum value of the energy function.

## 4. Experiment and Results

The data used in this study mainly come from the following aspects: questionnaire survey, interview, writing data before and after the test, and analysis of the final experimental results. All the data come from first-hand data, and the analysis methods are both qualitative and quantitative.

As can be seen in Table 1, the average number of lexical chunks used in the composition of the control class increased from 11.966 in the pretest to 12.031. However, the average number of lexical chunks used in the composition of the experimental class increased from 12.035 before the experiment to 16.068, with an increase of 33.5%.

The number of word pieces in the posttest composition of the experimental class is obviously more than that of the pretest composition, and it is also much larger than that of the posttest composition of the control class. It shows that in this experiment, ELL has obvious effect on enlarging the number of lexical chunks of students. Students can effectively input and store a large number of lexical chunks and generate them correctly and properly, which will make the writing language more accurate and true, make the text structure more coherent and logical, and effectively improve students' writing ability.

The rich vocabulary library enables students to successfully extract vocabulary in writing, which enhances students' interest in writing. The improvement of the awareness and requirements of using word fragments can significantly reduce students' dependence on grammar knowledge in writing, improve their self-confidence in writing, and increase their sense of accomplishment in learning English. After the experiment, students can consciously accumulate all kinds of relevant lexical chunks in combination with traditional recitation methods and strive to build a rich lexical chunk library and writing templates to make writing faster, smoother, and more effective.

According to the results of the paired *t*-test before and after the experimental class in Table 2, the effect of combining ELL with communicative competence has begun to appear. Reading and writing skills are helpful to some extent, which has improved students' comprehensive English ability and the overall English level of the class.

ELL is very important to improve students' enthusiasm for learning English, improve their vocabulary ability, and increase their vocabulary. First of all, students can understand each specific meaning of a word in a polysemous context and they can judge the cultural connotation of a word according to the context. Vocabulary is directly related to the language and cultural background, and the cultural background must be taken into account when learning and understanding words. All kinds of situational materials stimulate students' interest; they are more willing to participate in classroom activities and increase the interaction between teachers and students.

Through ELL, students change the way that they remember words by memorizing. They can better understand the meaning of words by using context clues, and on the basis of understanding, they can remember words according to the context. After teachers carry out ELL in class, students can improve their vocabulary learning methods and improve their ability to learn vocabulary independently by communicating with teachers and classmates.

In the existing research, few data-driven models can directly perform the task of predicting the difficulty of reading comprehension. This study evaluates the performance of the proposed model. The evaluation indexes are Pearson correlation coefficient and RMSE (root mean square error). The general experimental results of this model are shown in Figures 3 and 4.

The calculation difficulty of test questions is incomparable under different test questions, so the task of predicting the difficulty of practice questions should consider the statistical error of the content of test questions. Automatic reading task is different from the problem difficulty prediction task proposed in this paper. The model in this document can well understand the semantic information of the exercise text, and it is very helpful to predict the effect of the application task.

Test the performance of the cleaning tool based on Hadoop+Hive to clean 50G text call log data in different nodes to see if it has strong linear scalability. This paper thinks that this tool is absolutely linear and extensible. Generally speaking, the linear expansion ratio is only 1 in the theoretical case, so it is defined that when the linear expansion ratio is greater than 0.7, it proves that the tool has a large expansion capacity. The linear growth trend of Hive is shown in Figure 5.

It can be seen that when the number of computing nodes is increased to 10 times, 20 times, and 30 times of the original number of nodes, the performance gains are 3.95, 4.21, and 3.66, respectively, and the linear expansion indexes are 0.914, 0.928, and 0.93, respectively. It can be seen that the data cleaning tool based on Hadoop+Hive has excellent linear expansion. Therefore, in practical application, we can increase the overall mining speed by adding more computing resources. In practical application, the computing resources should be reasonably adjusted according to the running status of nodes, so as to avoid the critical point caused by the excessive growth of resources and unnecessary cost waste.

The paper evaluates the algorithm in terms of data volume and the number of computing nodes in order to confirm the model's scalability. It then discusses the DM results to highlight the significance of the DM results. 500000000 transactions are contained in 50G of data.  Figure 6 displays the outcome in full.

It can be seen that the calculation time of this model increases linearly with the increase of data volume, which shows that the Hadoop framework parallelizes data according to the data block size. With the increase of the number of nodes, the model in this paper has always maintained a high scalability, which shows that the model based on the Hadoop platform in this paper is very suitable for cloud computing applications and can greatly expand the generality result of effective computing on computing resources.

Through data cleaning of students' language learning achievements, 400 valid data were obtained, including students' four-dimensional achievements and ELL achievements. Pearson correlation coefficient is used to study the correlation between them. The scatter diagram of language achievement and ELL achievement is shown in Figure 7.

The school can therefore estimate the kids' results because there is a considerable association between the two. The learning scores can be reached at the highest ELL language level. The outcomes of students' thorough quality evaluations and their academic accomplishments diverge to some extent. Schools should promote students' holistic growth, which should be balanced in all facets aside from their academic accomplishments. In the West, cultural phenomena are a highly frequent occurrence in language studies. Nevertheless, a lot of people in today's society claim that English is a cohesive language. It is important to note that this is merely a surface-level phenomenon. English is more influenced by culture, according to the ELL study. For instance, using culture when applying English is prohibited. English has a strong linguistic allure since it is a historical language. We should be adept at sifting through the connotation and philosophical underpinnings of the language as we learn it.

In the process of language development, it can be seen that language is invented and created by human beings but language restricts human activities and this mutual restriction constantly promotes the development of linguistics. In recent years, the academic research on language and literature has been deepened but there are few works that really combine reality with innovation. Therefore, at this level, there is a very large perspective and research space. In the actual process of ELL research and analysis, we should make full use of cultural research methods and absorb the basic ideas and related ideas of English-speaking countries to the maximum extent. Teachers are required to spend more time and energy on the strict selection and evaluation of these materials when preparing lessons and even record microlessons when no suitable materials are found, so as to finally improve the teaching efficiency.

## 5. Conclusion

As an important means to cultivate students' language ability, ELL plays an important role in students' learning. We should change the old ideas and concepts, integrate multidimensional perspectives into ELL research, and create a good learning environment from the perspectives of cultural studies, philosophy, and politics, so as to fully stimulate students' enthusiasm for learning. From the results of the *t*-test, it can be seen that the comprehensive effect of ELL on communicative competence has begun to appear. Adopting the teaching method that focuses on the development of communicative competence in ELL is helpful to ELL, and students' comprehensive English ability has been improved to some extent. When the number of computing nodes is increased to 10, 20, and 30 times of the original number of nodes, the performance gains are 3.95, 4.21, and 3.66, respectively, and the linear expansion indexes are 0.914, 0.928, and 0.93, respectively. Hadoop+Hive's data cleaning tool has excellent linear scalability. Providing personalized learning services is of great significance to systematic enterprise management and students' learning effect.

## Figures and Tables

**Figure 1:** Framework model of the intelligent teaching system.

**Figure 2:** Distribution diagram of candidate set data nodes.

**Figure 3:** Pearson correlation coefficient of the model.

**Figure 4:** RMSE of the model.

**Figure 5:** Hive linear growth graph.

**Figure 6:** Test performance under 50G data.

**Figure 7:** Analysis of language achievement and ELL achievement.

**Table 1:** Comparison of lexical chunks before and after the test.

Classes	Total number of people	Pretest		Posttest	
		Mean value	Standard deviation	Mean value	Standard deviation
Experimental class	60	12.035	5.538	16.068	7.624
Control class	60	11.966	5.412	12.031	8.213

**Table 2:** The results of the paired *t*-test before and after the experimental class.

	*t*	Sig. (bilateral)
Pre-/postlistening test	−3.25	0.001
Grammar pretest/posttest	−4.41	0.000
Reading pretest/posttest	−5.52	0.000
Writing pretest/posttest	−3.09	0.002

## Data Availability

The data used to support the findings of this study are available from the corresponding author upon request.
